RETRACTED

# Role of Nutritional Support under Clinical Nursing Path on the Efficacy, Quality of Life, and Nutritional Status of Elderly Patients with Alzheimer's Disease

**DOI:** 10.1155/2022/9712330

**Published:** 2022-04-28

**Authors:** Haiyan Wu, Ya Wen, Saijin Guo

**Affiliations:** ^1^YongZhou Vocational Technical College, Yongzhou, Hunan Province, China; ^2^Emergency Department, Beijing Friendship Hospital Affiliated to Capital Medical University, Beijing, China

## Abstract

**Objective:**

To study the effect of nutritional support under the clinical nursing path on the nursing effect, quality of life, and nutritional status of elderly patients with Alzheimer's disease.

**Methods:**

110 elderly patients with Alzheimer's disease admitted to our hospital from February 2018 to October 2019 were randomly selected and assigned at a ratio of 1 : 1 via random draw to receive either routine nursing (control group) or nutritional support under the clinical nursing path (experimental group). Outcome measures included nursing efficiency, quality of life index (QLI) score, Pittsburgh sleep quality index (PSQI) score, Mental Status Scale in Non-psychiatric Settings (MSSNS) score, social disability screening schedule (SDSS) cognitive function score, and Mini Nutritional Assessment (MNA).

**Results:**

Nutritional support under the clinical nursing path was associated with significantly higher nursing efficiency and quality of life scores versus routine nursing (*P* < 0.05). Nutritional support under the clinical nursing path resulted in significantly lower PSQI, MSSNS, and SDSS scores, and fewer malnourished cases versus routine nursing (*P* < 0.05).

**Conclusion:**

Nutritional support under the clinical nursing pathway can significantly improve the quality of life, cognitive function, psychological status, and nutritional status of elderly patients with Alzheimer's disease, and has high application value.

## 1. Introduction

Alzheimer's disease is a mental illness with a high prevalence among the elderly. Its causes of onset can be mainly divided into degenerative brain diseases as the patient ages and encephalography elicited by the insufficient blood supply to the brain due to cerebrovascular disease [1–3]. There are currently no specific medications for Alzheimer's disease since it is an irreversible disease. Its imaging manifestations include widening of the cerebral sulcus and shrinking of the brain parenchyma, and its symptoms include a decline in memory, significant changes in personality, even dementia, and facial paralysis in severe cases [4–6]. The quality of life of patients with Alzheimer's disease is severely compromised, which also poses considerable psychological and economic pressure on their families. Clinical nursing for elderly patients with Alzheimer's disease is considered an effective method to alleviate the symptoms and delay disease onset. Studies showed that adequate daily nutrition for patients with Alzheimer's disease could significantly delay the onset, alleviate the symptoms, and further reduce the pressure on the patients and their families [7–9].

RETRACTED

The clinical nursing pathway is a process-oriented and rationalized nursing model. The use of the clinical nursing pathway in nutritional support for elderly AD patients to regularly screen and rate patients' nutritional risk and develop clinical care plans can achieve desirable nursing outcomes. The clinical care pathway can compensate for the randomness of conventional care with little dependence on clinical experience and theoretical knowledge of clinical nurses. Nutritional support under the clinical nursing pathway can improve the nutritional status of AD patients, enhance their organism immunity, and improve their quality of life.

In the present study, elderly patients with Alzheimer's disease were recruited to study the effect of nutritional support on the quality of life, mental condition, and cognitive functions of elderly patients with Alzheimer's disease. The specific study is reported as follows.

The innovation of this study lies in the combination of nutritional support given under the clinical care pathway to compensate for the shortcomings of conventional care, but the limitation of this study is the absence of long-term follow-up data and the lack of clinical data on the psychological and physiological aspects of patients' long-term care.

## 2. Data and Methods

### 2.1. Ethical Statement

The study was approved by the Ethics Committee of Beijing Friendship Hospital, and the patients and their families were informed of the purpose and process of the experimental study and signed the informed consent. The ethics approval number was 2017-11-29.

### 2.2. General Data

A total of 110 elderly patients with Alzheimer's disease admitted to our hospital from February 2018 to October 2019 were assigned at a ratio of 1 : 1 via random draw to a control group or an experimental group. The age of the patients in the experimental group ranged from 60 to 83 years, while the age of the patients in the control group ranged from 60 to 85 years. The two groups showed similar baseline data (*P* > 0.05).

### 2.3. Inclusion/Exclusion Criteria

#### 2.3.1. Inclusion Criteria

① In line with the imaging and clinical symptoms of Alzheimer's disease
② Aged ≥60 years old
③ No history of drug allergy, no history of drug abuse, and no bad habits
④ With no other organic diseases; with normal functions of the heart, lung, and kidney
⑤ This study was approved by the hospital ethics committee, and all patients participated and signed the informed consent form voluntarily.

RETRACTED

### 2.4. Exclusion Criteria

① With severe cardiovascular and cerebrovascular diseases or received relevant surgical treatment
② With major surgical treatment recently
③ Patients or their families refused to participate in this study.

### 2.5. Methods

The control group was treated with routine clinical nursing, including the development of nursing plans based on the patient's symptoms, health education on the disease and treatment for the patients and their families, and psychological counseling. The experimental group was treated with nutritional support plus routine nursing (same as the control group). A nutrition intervention pathway consists of three components: core support, intensive care, and enhanced care. (1) Targeted nutritional support was provided according to the patient's nutritional status. (2) The patient's diet was based on the basic principles of coarse grains, supplemented by fine grains, less meat, more vegetables, low salt and sugar, small meals for a day-long stream, and a reasonable combination of nutrition. (3) A glass of honey or salty water was provided every morning to activate the intestines. (4) Adequate daily intake of protein and vitamins was ensured. (5) The specific diet composition can refer to the Mediterranean diet [10–12]. The daily intake of fat and sugar was reduced for obese patients, and the nutrient intake was increased for patients with excessive weight loss and malnutrition. The patients and their families were educated about nutritional support.

### 2.6. Outcome Measures

Outcome measures included the efficacy of nursing, the quality of life index (QLI) score [13], Pittsburgh sleep quality index (PSQI) [14], the Mental Status Scale in Non-psychiatric Settings (MSSNS) scores [15], social disability screening schedule (SDSS) scores [16], and also malnutrition status which was assessed by Mini Nutritional Assessment (MNA) [17]. Nursing efficacy: Markedly effective: the patient showed a stable condition and good nutritional status, quality of life, and psychological state during the nursing. Effective: the patient's memory and cognitive function saw a decline, the nutritional status remained normal, and the quality of life and psychological state were relatively stable during the nursing process. Ineffective: the patient's condition was aggravated with severe malnutrition or overnutrition, and their quality of life and psychological status were poor during the nursing process.

RETRACTED

QLI includes rating criteria for daily routines, work and life, and interpersonal relationships. The score of each dimension is 10 points. The higher the score, the better the quality of life. The scale PSQI is ranged from 0 to 21 points. The higher the score, the worse the sleep quality. For the MSSNS, the rating of 60 points serves as the standard of differentiation. Any rating lower than 60 indicates a normal mental state; any rating between 60 and 70 indicates a mildly abnormal mental state; any rating above 70 indicates an abnormal mental state.

The SDSS is ranged from 0 to 20 points. The higher the score, the lower the cognitive function. The scale of malnutrition status assessed by the mini nutritional assessment (MNA), is ranged from 0 to 30 points. A score higher than 23.5 points indicates a good nutrition status; a score between 17 and 23.5 points indicates a moderate malnutrition status; a score less than 17 points indicates a severe malnutrition status.

### 2.7. Statistical Analysis

All the information and data in this study were processed and analysed using the statistical software SPSS21.0. The measurement data were expressed in form of ($\bar{x}$± *s*) and examined using a *t*-test. The counting data were expressed in (*n* (%)) and examined for differences using the X^2^ test. Significance was claimed at a *P* value of <0.05.

## 3. Results

### 3.1. Baseline Data

The two groups showed similar baseline data (*P* > 0.05) (Table 1).

### 3.2. Nursing Efficacy

Nutritional support under the clinical nursing path was associated with a higher nursing efficacy versus routine nursing (*P* < 0.05). (Table 2).

### 3.3. QLI Scores

The scores of daily activities, work and life, and interpersonal relationships on the quality of life scale were significantly higher in the experimental group than in the control group (*P* < 0.05). (Figure 1).

### 3.4. PSQI and SDSS

Nutritional support under the clinical nursing path resulted in significantly lower scores of PSQI and SDSS versus routine nursing (*P* < 0.05) (Table 3).

### 3.5. MSSNS

The patients receiving nutritional support under the clinical nursing path showed a significantly lower MSSNS score versus routine nursing (*P* < 0.05) (Figure 2).

### 3.6. Malnutrition Status

Nutritional support under the clinical nursing path resulted in a significantly lower incidence of malnutrition (10.9%) status versus routine nursing (41.89%) (*P* < 0.05). (Table 4).

## 4. Discussion

Reduced vascular elasticity in the elderly predisposes to the development of atherosclerosis and consequently cardiovascular and cerebrovascular diseases. A common cause of Alzheimer's disease is encephalanalosis caused by the long-term insufficient blood supply to the brain due to cardiovascular and cerebrovascular diseases [13, 14]. Neurodegenerative disease is also considered a pathogenic factor [15–17]. The etiology of Alzheimer's disease is elusive and no specific medicines are available currently, which has caused great difficulties in the clinical treatment of Alzheimer's disease. The disease is irreversible and its general symptoms include a decline in memory, significant changes in personality, gradual loss of ability to perform daily routines, a decline in social communication ability, and decline in intelligence [18, 19]. It has been reported that healthy and reasonable living habits can prevent or delay the onset of Alzheimer's disease. Healthy living habits include a reasonable diet composition, a good daily schedule, exercise habits, and engagement in intellectual activities.

RETRACTED

The evaluation standard of nursing efficacy shows that nursing efficacy is of great relevance to the nutritional status, quality of life, and mental state of patients. The results of the present study showed that nutritional support under the clinical nursing path was associated with a significantly higher nursing efficiency versus routine nursing, indicating that nutritional support can improve the quality of life, mental state, and nutritional status of patients, which was evidenced by the higher QLI score in patients receiving nutritional support under the clinical nursing path in the present study.

The research results by Liu et al. [20] showed a similar outcome. In her study, nutritional support under the clinical nursing path resulted in significantly higher quality of life scores and fewer malnourished cases. Additionally, nutritional support under the clinical nursing path in the present study was associated with significantly lower scores of PSQI, MSSNS, and SDSS versus routine nursing (*P* < 0.05), suggesting that nutritional support can significantly improve sleep quality, mental state, and cognitive function of patients with Alzheimer's disease.

The status of malnutrition in the two groups was assessed by MNA, and the results in the present study demonstrated fewer malnourished cases in the experimental group versus the control group (6 vs. 23), indicating that nutritional support can maintain a good nutritional status of Alzheimer's patients and alleviate the condition of illness.

In traditional Chinese medicine (TCM), the brain is the center of the spirit and the basis of spiritual memory. The loss of essence and blood in the elderly, the emptiness of the brain marrow, and the gradual loss of memory will lead to symptoms such as sluggishness and forgetfulness. The brain is closely related to the kidney, as the brain is the center of marrow, and the marrow is produced in the kidney through the harmonization of Yin and Yang. External disturbances can lead to dysfunction of the internal organs, malfunction of qi and blood, and blood stasis, which blocks the brain circulation, deprives the marrow sea of nourishment, and disables mental and spiritual functions. The common symptoms of AD patients with deficiency of kidney essence and internal obstruction of blood stasis include white hair, loss of teeth, nocturnal urination, obscured eyes, purple tongue, and astringent pulse. In Practical Blood Stasis Evidence, it is mentioned that the clinical manifestations of AD with kidney deficiency and blood stasis are progressive decline in memory, mental fogginess, slow thinking, poor calculation, disorientation, pale purple tongue, and sunken and weak pulse. This indicates that the primary symptom of AD blood stasis patients is memory loss, followed by cognitive decline and decreased ability to perform activities of daily living, which requires more attention from healthcare professionals. Currently, most of the TCM interventions for AD blood stasis are focused on the improvement of patients' memory, cognitive function, and activities of daily living. Memory loss compromises patients' ability to perform activities of daily living and reduces their quality of life; so, many TCM researchers have conducted clinical or basic research on the early symptoms of blood stasis in AD and achieved favorable results.

RETRACTED

Abnormal *β*-amyloid deposition is the core link in the pathogenesis of AD, and plays a leading role in the occurrence and development of AD. *β*-amyloid is a small molecular polypeptide composed of 39–43 amino acids, and it is derived from the hydrolysis of amyloid precursor protein (APP). APP is the precursor protein of *β*-amyloid, and mutation and overexpression of the APP gene can cause the overproduction of *β*-amyloid in vivo. Icariin can reduce the expression level of APP in the hippocampus of APPV717I transgenic mice and reduce the amount of *β*-amyloid. The active ingredient bibuminine/dihydrobibuminine (1 : 0.8) can effectively inhibit the expression of APP mRNA and protein in SK-N-SH cells at the same time, thereby reducing the production of *β*-amyloid. Berberine igAPP-mutant mice can reduce the phosphorylation level of APP by inhibiting the activity of glycogen synthase kinase (GSK3), further reduce the generation of *β*-CTF through the AKT/GSK3*β* signaling pathway, and reduce the soluble and production of insoluble beta-amyloid. The immature APP is N-linked glycosylation on the endoplasmic reticulum and then matures after subsequent processing such as in the Golgi apparatus. In a variety of cells stably transfected with APP751, it has been proved that curcumin can affect the processing and modification of immature APP in the endoplasmic reticulum, delay the maturation of APP, and reduce the level of *β*-amyloid.

RETRACTED

## 5. Conclusion

Nutritional support is a preferred method in elderly patients with Alzheimer's disease with respect to its strength in improving the quality of life and nursing efficacy rate, improving the quality of sleep, mental state, cognitive function, and nutritional status of patients.

## Figures and Tables

**Figure 1:** Comparison of QLI between two groups. The abscissas, from left to right, represent the indicators of the experimental group and the control group in the QLI, which are daily routines, work and life, and interpersonal relationships. While the ordinates represent the QLI points. ^∗^represents that daily routines points (8.26 ± 1.57) of the experimental group was compared with the daily routines points (6.00 ± 1.04) of the control group. *t* = 8.90, *P* < 0.001. The difference is statistically significant; ^∗∗^represents that the work and life points (9.03 ± 0.51) of the experimental group was compared with the points (6.27 ± 1.04) of the control group. *t* = 10.87, *P* < 0.001. The difference is statistically significant; ^∗∗∗^represents the interpersonal relationship points (8.16 ± 1.13) of the experimental group was compared with the interpersonal relationship points (5.77 ± 1.25) of the control group. *t* = 10.52, *P* < 0.001. The difference is statistically significant.

**Figure 2:** Comparison of the MSSNS of the two groups. The abscissas represent the experimental group and the control group from left to right, and the ordinates represent the MSSNS points. ^∗^represents that the MSSNS points (51.68 ± 5.22) of the experimental group were compared with the MSSNS points (56.38 ± 5.09) of the control group. *t* = 4.78, *P* < 0.001. The difference is statistically significant.

**Table 1:** Statistics of general data comparison ($\bar{x}$ ± *s*).

Group	Experimental group	Control group	t/*X*2	*P* value
Gender (male/female)	32/23	30/25	0.15	0.70
Age (years)	76.05 ± 4.24	75.83 ± 5.11	0.25	0.81
Height (cm)	163.18 ± 10.54	162.92 ± 10.88	0.13	0.90
Weight (kg)	70.25 ± 8.22	69.77 ± 8.51	0.30	0.76
Course of disease (years)	3.86 ± 1.52	3.90 ± 1.67	0.13	0.90
History of smoking (years)	13.51 ± 3.33	13.96 ± 3.67	0.67	0.50
History of drinking (years)	20.83 ± 4.09	20.07 ± 3.96	0.99	0.32
Hypertension (case)	9	10	0.06	0.80
Diabetes (case	7	10	0.63	0.43
Hypertension (case)	10	8	0.27	0.61

**Table 2:** Comparison of the efficacy rate of nursing.

Group	Markedly effective	Effective	Ineffective	Total efficacy rate (%)
Experimental group	35	13	7	87.27%
Control group	14	21	20	63.64%
X^2^				8.30
*P* value				0.004

RETRACTED

**Table 3:** Comparison of the PSQI and SDSS between the two groups ($\bar{x}$ ± *s*, points).

Group	PSQI ($\bar{x}$ ± *s*, points	SDSS ($\bar{x}$ ± *s*, points)
Experimental group	10.36 ± 2.06	9.84 ± 2.91
Control group	15.27 ± 3.38	16.53 ± 4.41
t	9.20	9.39
*P* value	<0.001	<0.001

**Table 4:** Comparison of malnutrition status.

Group	Good nutritional status	Moderate malnutrition	Severe malnutrition	Occurrence rate of malnutrition
Experimental group	49	6	0	10.90%
Control group	32	16	7	41.82%
X^2^				13.53
*P* value				<0.001

## Data Availability

The datasets used and analysed during the current study are available from the corresponding author on reasonable request.
